# Evaluation of Salt Tolerance Mechanism and Study on Salt Tolerance Relationship of Different Salt-Tolerant Wheat Varieties

**DOI:** 10.1155/2022/2395568

**Published:** 2022-10-05

**Authors:** Weiwei Wang, Yong Zhao, Wei Wang, Ke Xu, Liya Niu, Liang Yu, Jing wei Zou, Zhi Wang, Yu jie Zhang, Fengzhi Wang, Shuhua Zhang, Xueju Yang

**Affiliations:** ^1^College of Agronomy, Hebei Agricultural University, Hebei Baoding 071000, China; ^2^Cangzhou Academy of Agriculture and Forestry Sciences / Hebei Key Laboratory of Crop Salt-Alkali Tolerance Evaluation and Genetic Improvement, Hebei Cangzhou 061001, China; ^3^College of Life Science, Hebei Agricultural University, Hebei Baoding 071000, China

## Abstract

The physiological and biochemical indexes of different salt-tolerant wheat cultivars under salt stress are affected to different degrees. The changes in physiological and biochemical indexes in salt-tolerant wheat varieties are moderate, while salt-sensitive wheat varieties have bigger changes. In this article, through comprehensive utilization of germination and seedling indoor test morphological indexes, physiological and biochemical index, and output index, combined with the evaluation mechanism of wheat's salt resistance, different salt tolerance types in the middle and lower reaches of the Yangtze River in Shandong province were studied; a collection of 100 wheat varieties and 11 wheat varieties planted over a large area were classified into three groups: strong salt resistance, medium salt resistance, and weak salt resistance. Comparative analysis of different wheat varieties' salt resistance evaluation mechanism was performed, as well as the analysis of the germination rate of wheat varieties, coleoptile growth situation, emergence rate, protect wheat seeding rate, tillering rate, seedling height, root length, seedling dry weight, wet weight, number of leaves, plant growth situation, agronomic characters of the Na^+^/K^+^ ratio, and other physiological and biochemical indexes such as salt resistance index. The evaluation mechanism of salt tolerance and the relationship of salt tolerance of different wheat varieties were obtained. The results showed that there were significant differences in salt tolerance among the 100 wheat varieties at the germination stage. Among them, three varieties, YM (Yangmai) 25, YM (Yangmai) 24, and EM (Emai) 25, had the strongest salt tolerance at the germination stage, reaching the level of the salt tolerance variety DK 961, and the salt tolerance was in the first level, while NM 17, NM 23, and other 21 varieties reached the level of the salt tolerance. These 24 varieties with strong salt tolerance at the germination stage can be used to screen the salt tolerance of wheat planted in the saline soil of Jiangsu coastal beach.

## 1. Information

Saline-alkali land is widely distributed in Africa, Asia, Oceania, and South America. At present, the global land salinization area is around 954 million hm^2^, accounting for 7% of the global land area, and this number is still rising. The national soil survey shows that the saline-alkali land covers an area of around 99.13 million hm^2^, accounting for 10% of the available area in China, among which the salinized land in cultivated land accounts for 6.62% of the cultivated land area in China, which is around 9.209 million hm^2^ [1]. Due to the harm caused by human activities, the area of secondary saline-alkali land is also increasing. Due to the high salt content and alkalinity of saline-alkali land, the poor soil structure and the lack of nutrients seriously affect the growth and development of plants, which mainly manifests as osmotic stress. Salt stress will inhibit the growth and differentiation of tissues and organs, reduce the ability of plants to absorb water and nutrients, reduce the number of leaves, reduce leaf area, decrease chlorophyll content, and then affect photosynthesis, resulting in lower plant yield [2]. Ion toxicity can occur in plants: salt stress conditions, plants with Na^+^/K^+^ ratio, and high Na^+^ damage to the membrane's protective enzyme system cause the peroxidation of the membrane system and membrane permeability; K^+^ and Ca^2+^ ion exosmosis leads to ionic imbalance in the plant body, causing cell water difficulties, such as water stress and physiological drought of plants. Oxidative stress can also occur: salt stress increases the reactive oxygen species in the body and the lipid peroxidation of the cell membrane, thus causing the destruction of the structure and function of the cell membrane and the selective loss of the membrane, leading to a series of physiological and metabolic disorders affecting the growth and development of plants [3, 4]. Wheat yield is low, so it is necessary to plant wheat varieties with salt tolerance. Salinity tolerance of crops is an extremely complex trait, which is easily affected by environmental conditions. In the growth cycle of crops, the salt tolerance is different at different developmental stages. Previous studies have suggested that the early development of crops lays the foundation for the whole growth cycle, and the early stress damage has a great influence on the later growth and the final yield. Therefore, the germination stage in the early stage of crop development is an important period for crop salt tolerance research. There were significant differences in salt tolerance among wheat cultivars, especially in the early germination stage.

In recent years, some scholars at home and abroad have studied the salt tolerance of wheat during germination. Nakayama et al. conducted RNA sequencing of roots of three strains of salt-tolerant hexaploid wheat, salt-tolerant common wheat, and salt-sensitive common wheat, and the results showed that the synthetic hexaploid wheat had salt tolerance mechanisms that common wheat did not have, which might be potential breeding material for salt tolerance [5]. Zhang et al. applied salt stress on 293 wheat germplasm at the germination stage and selected 16 germplasm with high salt tolerance at the germination stage [6]. Zhangtingting et al. identified 30 spring wheat varieties (lines) for salinity tolerance at the germination stage and screened out 7 varieties with high salinity tolerance at the germination stage [7]. Peng et al. screened 328 wheat materials and selected 21 materials with high salt tolerance at the germination stage [8]. New salt-tolerant wheat varieties provide excellent materials. Liu Xu et al. identified and screened 11 wheat varieties with strong salt tolerance by conducting salt tolerance tests on 400 wheat varieties at the bud stage and seedling stage: “Red Hornhopper,” “Keyi 26,” “Hope,” 98-46, 98-113, 98-131, 98-160, 98-161, 98-163, etc. Among them, the salt tolerance of 98-113 and 98-160 wheat is the most prominent [9]. Zhang Qiaofeng et al. treated 293 wheat germplasm with salt stress at the bud stage and seedling stage, and screened five new salt-tolerant germplasm: Marmin-Minhardi × H44-Minturki, white husk wheat, Huashu Pui, Shenmai, and Top seed hammer. Gong Wenping et al. identified the salt tolerance of 417 wheat materials selected from the International Maize and Wheat Improvement Center (CIMMYT), and selected four wheat salt tolerance germplasm, CM58, CM163, CM439, and CM440 [10]. Guo et al. selected Hitch, TVTOPL-9, and Xinong 509 cultivars with high salt tolerance by identifying the salt tolerance of some American wheat germplasm resources [11]. Ma and Weng identified the salt tolerance of 28 spring wheat germplasm from the United States at the bud stage and seedling stage, and showed SW10 and SW12 germplasm had high salt tolerance values for promotion [12]. Guo et al. used different salt stress concentrations to identify the salt tolerance of 161 wheat samples from Tibet at the seedling stage, and selected 14 salt-tolerant materials, among which three were not sensitive to the salt stress concentration gradient [13]. Through salt stress treatment and salt tolerance identification of three wheat mutants, Qiao et al. found that CAO8113K had high salt tolerance [14]. Li identified 13 wheat varieties such as Ningchun 4, Ningchun 16, Ningchun 20, and 98XW series on saline-alkali soil, among which Ningchun 16, Jing3377, and salt-tolerant barley showed high salt tolerance [15]. In addition, there are some salt-tolerant varieties: the salt-tolerant and high-yield wheat varieties SR3, XX12, Chahdianhong, etc., developed by asymmetric somatic cell fusion technology.

Based on the evaluation method of salt tolerance adopted by Yu Guihong, the method adopted by Gong [16], and the evaluation method of salt tolerance in the standard, this paper compared and analyzed the evaluation mechanism of salt tolerance of different wheat varieties. Through the analysis of the germination rate of wheat varieties, coleoptile growth situation, emergence rate, protect wheat seeding rate, tillering rate, seedling height, root length, seedling dry weight, wet weight, number of leaves, plant growth situation, agronomic characters of Na^+/^K^+^ ratio, and other physiological and biochemical indexes such as salt resistance index of different varieties of wheat salt resistance, the evaluation mechanism and the relationship with salt resistance were studied.

## 2. Test Protocol

### 2.1. Test Materials

A total of 100 wheat varieties collected from wheat areas in the middle and lower reaches of the Yangtze River and 11 wheat varieties with large extended planting areas in Shandong Province were selected for salt-tolerant germplasm. The varieties widely grown in Shandong were DK(DK) 961, JM(JM) 22, QM(QM) 6, YN(YN) 24, Lumai(LM) 21, LX(LX) 99, YN(YN) 836, QF(QF) 1, TN(TN) 18, SN(SN) 21, and YN(YN) 21,100, as shown in Table 1.

### 2.2. Test Scheme

#### 2.2.1. Salt Stress Test in Wheat Germination

This experiment was carried out in the cultivation room. 100 full and neat wheat grains of each variety were selected, sterilized with 75% alcohol solution for 5 min, rinsed several times with deionized water, evenly placed on the wheat germinating box (the length and width of the germinating box were 12 cm), and covered with three layers of filter paper. The cultures were incubated in NaCl solution incubators with 5 concentration gradients of 80, 160, 240, 320, and 400 mmol/L. During the incubation period, 15 ml salt solution was added to each box, and 15 ml distilled water was used instead of salt solution in the control group. Three replicates were set for each treatment, and the constant illuminance at 25°C was unchanged. Plants were randomly selected for the determination of relevant morphological indexes (demonstrated in Figure 1).

#### 2.2.2. Salt Stress Test at the Seedling Stage

This experiment was carried out in the cultivation room. After the germination stage test, 7 wheat varieties with different salt tolerances, NM15, YM22, EM12, JM 22, QM 6, DK 961, and QF 1, were selected. After incubation with distilled water for 24h in a constant temperature light incubator at 25°C with dewlap, the grains with uniform and consistent de were selected and cultured with Hoagland nutrient solution. The culture method was oxygen culture. The seedlings were cultured in 1/2 Hoagland nutrient solution for the first week after uniform emergence and were then changed to Hoagland total nutrient solution after one week of growth. The roots of wheat were washed at the seedling stage with the same growth, and the treatments were changed to nutrient solutions with different NaCl concentrations; the concentration gradients were 80, 160, and 240 mmol/L stress nutrient solution, respectively. The control was cultured with nutrient solution, and the experiment for each variety was repeated three times. Leaves and roots of plants were randomly selected for the determination of physiological, biochemical, and osmotic ions. In this experiment, the hydroponics method was used to identify salt tolerance in the wheat seedling stage. The specific steps were as follows:

1. First, the prep work was done: 1% hydrogen peroxide was prepared, the Petri dishes were washed an sterilized, the PCR plates to be used were prepared, and the incubator was sterilized with 70% alcohol.
2. Wheat seeds with full grain and no damage were selected, sterilized with 1% hydrogen peroxide, and placed in a Petri dish covered with qualitative filter paper. The seeds were placed in the Petri dish with tweezers. Water was added to the Petri dish to wet the qualitative filter paper; finally, the Petri dishes were placed in an incubator at 24°C for cultivation, and purified water was added to the dishes regularly to keep the qualitative filter paper moist.
3. The material number was marked on the PCR plate. When the seed root grew to 2-3 cm, the seeds with the same growth trend were selected and transferred to the prepared PCR plate. The PCR plate was placed into 0.8 g/ml nutrient solution (ensuring that the root was immersed in the nutrient solution); the experimental conditions were as follows: the photoperiod was 16 h/24°C in light and 8 h/16°C in darkness, and the water was changed once every two days to prevent mildew. Salt stress began when it grew to two leaves.
4. 0.8 g·m/L nutrient solution with NaCl concentrations of 80, 160, and 240 mmol/L was prepared. The wheat grown to two leaves was put into the salt solution and grown in an incubator, with the water being changed every two days.

## 3. Determine the Item

### 3.1. Determination of Morphological Indexes Related to the Germination Test

Coleoptile length and germination potential were measured on the 3rd day (72 h) of germination. On the 7th day of culture (168 h), the number of germinated seeds was investigated, the germination rate was calculated, the longest root length of seeds and seedling height were measured, and the number of seed roots and the fresh weight of seedlings were recorded, and the growth rate of the first leaf was observed and recorded from the 7th day (168 h).

### 3.2. Field Sample Sampling Method

 During the flowering period of wheat, 200 wheat plants with the same day of flowering and basically the same growth without pests and diseases were selected for each treatment to be labeled, and wheat plants were taken from the labeled wheat every 7 d from the flowering period, and 20–25 wiped wheat flag leaves were cut and stored in the ultra-low temperature refrigerator by liquid nitrogen treatment for measurement of wheat physiological and biochemical indexes. The cob with uniform size and uniform growth was selected; 10 ears were sampled for each treatment, and 10 grains of the central cob were taken for each ear. The cob was dried at 105°C for 30 min and then dried at 80°C to constant weight. The dry weight was converted into 1000-grain weight to calculate the grain filling efficiency. Before maturity, a complete 1 m^2^ panicle number was selected from each plot, which was converted into panicle number per unit area. At maturity, 10 intact plants were selected from each plot. After harvesting, the number of grains per ear was obtained using the seed test, and the 1000-grain weight was determined by threshing after air drying. Finally, it was converted into terms of yield.

### 3.3. Determination of Wheat Leaf Senescence and Osmotic Regulatory Substances

1.5 g sample was cut into pieces and added to 15 ml 150 mM phosphate buffer with a pH value of 7.0, ground in the ice bath, frozen and centrifuged at 15,000 ×g for 5 min, and the supernatant was the crude extract of the enzyme for the determination of MDA, SOD, and POD.

### 3.4. Determination of Seedling Root Activity

0.2 g of the sample to be tested was weighed, and 2 ml of 1%TTC, 5 ml of 0.1 m phosphate buffer, and 3 ml of distilled water were added and held at 37°C for 1 h; then, 2 ml of 1 M sulfuric acid was added to terminate the reaction, the roots were removed, the water was absorbed, the sample was ground, the homogenate was transferred to a funnel and filtered into a 10-ml test tube, and the volume was fixed to 10 ml with eTOAC as a blank control. The optical density was measured at 485 nm, and the TTC reduction amount was obtained by checking the standard curve.

### 3.5. Ion Extraction and Determination Methods

In the seedling stage of the experiment, 10 plants were randomly selected from each treatment, rinsed repeatedly with deionized water, dried with absorbent paper at 105°C for 30 min, dried at 80°C to constant weight, and ground into powder. 200 mg was accurately weighed, and 12 ml of concentrated nitric acid and perchloric acid in the proportion of 5 : 1 were boiled and extracted in an eliminative furnace for 4 h; then, the volume was fixed to 10 ml. The contents of Na^+^, K^+^, and Ca^2+^ were determined using the PE Optima 8000 atomic absorption spectrophotometer.

### 3.6. Determination of Photosynthetic Characteristics of Flag Leaves

During the flowering stage of winter wheat, the flag leaf tags of the plants with the same growth were selected for each treatment. From the flowering stage, the SPAD-502 chlorophyll meter made in Japan was used to measure the chlorophyll content from 1/3 of the leaf tip every 7 days from 9:00 to 11:00 in the morning without wind, and the SPAD value was used to represent the chlorophyll content. Ten wheat flag leaves were randomly selected from each row for the determination of chlorophyll content, and the average was recorded. The net photosynthetic rate (Pn), stomatal conductance (Gs), intercellular carbon dioxide concentration (Ci), and transpiration rate (Tr) of the flag leaf were measured using a LI-6400 photosynthetic apparatus (manufactured by Li-Cor, USA). Five leaves were measured in each replicate. In the flowering stage, 10 representative plants were selected from each plot, and all the leaves were cut off. The leaf area was measured using a LI-3100 leaf area meter, and LAI was calculated and measured every 7 days.

### 3.7. Methods for Determination of Wheat Yield and Yield Components

Before maturity, a complete 1 m^2^ panicle number was selected from each plot to check the panicle number in a hectare. At maturity, 10 intact plants were selected from each plot. After harvesting, the number of grains per ear was obtained by the seed test, and the 1000-grain weight was determined by threshing after air drying. Finally, it was converted into yield.

### 3.8. Data Analysis

Microsoft Excel 2019 and Origin 2022b were used to process and plot the test data. DPS7.05 statistical software was used to analyze the data and test the significance of the difference.

## 4. Evaluation Method of Salt Tolerance

### 4.1. Evaluation Criteria for Salinity Tolerance at the Germination Stage

According to the salt damage index proposed in the technical specification, the salt tolerance of wheat at the germination stage was graded and evaluated (as demonstrated in Figure 2).

(1) $$\begin{array}{c} \text{Salt damage index}=\frac{\left[\text{control germination rate}-\text{treatment germination rate}\right]}{\text{control germination rate}}\times 100\%. \end{array}$$

### 4.2. Evaluation Method of Wheat Leaf Senescence and Osmotic Regulatory Substances

The content of malondialdehyde (MDA) was determined according to the method used by Lin Zhifang. The activity of superoxide dismutase (SOD) was recorded according to Wang Aiguo's method. The activity of peroxidase (POD) was determined using the guaiacol colorimetric method. Peroxidase acted on o-methoxyphenol to produce brown-red tetra-methoxyphenol, with a characteristic absorption peak at 470 nm. Peroxidase activity was determined indirectly by measuring the content of tetra-methoxyphenol. The content of soluble protein was determined by the Coomassie brilliant blue method. The standard curve of bovine serum protein was plotted. The content of the proline was determined by the sulfosalicylic acid method. The soluble sugar content was determined by the anthrone colorimetric method.

### 4.3. The Limited Sodium Ability Evaluation of Wheat

According to Ref. [17], ability to limit sodium (Na^+^) = underground part content of Na^+^/Na^+^ content on the ground.

### 4.4. Comprehensive Evaluation of Salt Tolerance

Salt tolerance of crops is the overall performance of various crops in response to salt stress. There are differences in the mechanisms of salt stress adaptation among different crops. At present, there are various evaluation methods for wheat salt tolerance, including single-index analysis and multiple-index comprehensive analysis. Single-index analysis is mainly used to evaluate the salt tolerance of plants by calculating and analyzing the relative salt damage rate, which is suitable for screening the primary salt tolerance of a large number of materials. These methods are simple and rapid but ignore the differences in physiological morphological indexes such as plant height, root length, and osmotic potential in response to salt stress, and their results are one-sided. The comprehensive analysis of multiple indicators includes correlation analysis, membership function analysis, principal component analysis, principal component assignment weight reweighting method, regression analysis, and path analysis. This method can fully reflect salt tolerance from various aspects by analyzing multiple indicators at the same time. The comprehensive evaluation of plant salt tolerance by multivariate analysis can supplement the one-sidedness of single-element evaluation of plant salt tolerance to improve the accuracy of evaluation. It is scientific and reasonable to use multiple-index systems to evaluate the salt tolerance of plants.

## 5. Results and Analysis

### 5.1. Effects of Salt Stress on Relevant Indexes of Different Wheat Varieties during Germination

The salt tolerance test at the germination stage is the basis for the early identification of salt tolerance and the early selection of salt-tolerant individuals and varieties in wheat. The results showed that different wheat varieties showed consistent salt tolerance under salt stress, such as germination percentage, germination potential, root length, coleoptile length, seedling height, the growth rate of the first leaf, and seedling fresh weight. DK 961 and QM 6 showed high salt tolerance. YN 24, LX 99, QF 1, TN 18, and SN 21 showed moderate tolerance to salt stress. YN 21, LM21, YN 836, and JM 22 were sensitive to salt stress and had low salt tolerance.

The results showed that the relative values of germination percentage, germination potential, coleoptile length, root length, seedling height, the growth rate of the first leaf, and seedling fresh weight of 11 winter wheat varieties were significantly decreased, and there were significant differences among different varieties and concentrations. This is consistent with the research results of Ding [18], Ye [19], and Zhao [20] on the salt tolerance of wheat during germination. Considering the performance of each variety under different concentrations, the salt solution concentration reached 320 mmol/L, which was considered a high salt concentration stress, and winter wheat was difficult to grow. Multiple comparison results showed that the reduction range of each index was small under low salt concentration stress. However, when the salt concentration reached above 320 mmol/L, the indexes decreased sharply, especially in the salt-sensitive varieties. JM 22 and other cultivars could not germinate under high salt concentrations, and most cultivars could not extract the first leaf under high salt concentrations, indicating that winter wheat is not suitable for growth and development under high salt concentrations. The threshold of wheat salt tolerance concentration should be combined with wheat yield and other factors for subsequent studies. The root number of winter wheat during germination did not change regularly in the same variety under different concentrations or different varieties under the same salt concentration. The response of root number to salt stress was as follows: at higher salt stress concentration, the tested varieties still maintained more root number, which may be higher than the performance value on both sides of the concentration. This again indicates that salt stress has little effect on the root number of wheat, which is consistent with the study results of Li [21] using compound salt and Li et al. using NaCl single salt on wheat stress, indicating that the root number cannot be used as an index for the identification of salt tolerance at germination stage. However, the identification of salt tolerance of the wheat variety system requires further comprehensive studies on the physiological and molecular mechanisms of wheat during the whole growth period.

According to the technical specification of wheat salt tolerance identification and evaluation, the 11 winter wheat varieties, DK 961, and QM 6 had the strongest salt tolerance. Seven physiological traits, germination rate, germination potential, coleoptile length, root length, seedling height, the growth rate of the first leaf, and seedling fresh weight, can be used as effective indicators for indoor screening of winter wheat's germination stage (Figure 3).

### 5.2. Effects of Salt Stress on Osmotic Regulatory Substances and Root Activity of Wheat Seedlings

Studies have shown that increasing the activity of antioxidant enzymes and accumulating osmotic regulatory substances are the two most important mechanisms for plants to survive in an adverse environment. Antioxidant enzymes are a set of reactive oxygen species scavenging systems in plants, which can maintain the metabolism level of reactive oxygen species and maintain the structure and function of the membrane. The antioxidant enzyme system includes a series of enzymes, among which SOD is an important enzyme to scavenge oxygen free-radicals, mainly superoxide anion free-radicals. After salt stress treatment, salt-tolerant varieties could maintain relatively higher SOD activity than non-salt-tolerant varieties, which weakened membrane lipid peroxidation and alleviated salt stress damage to the membrane. The results showed that the SOD activity of the wheat seedling stage decreased with the increase in salt concentration. The SOD activity of QM 6 and DK 961 leaves decreased slightly with the increase in salt concentration and stress time, while the SOD activity of JM 22 and QF 1 decreased greatly. Salt stress caused a decrease in the SOD activity of wheat. POD can remove H_2_O_2_ produced by stress and is a member of the antioxidant enzyme system. He [22] believed that the POD activity of wheat under salt stress increased with the increase of salt concentration, but there were differences among varieties, and salt-tolerant varieties were higher than sensitive varieties. This study found that under salt stress, the varieties of wheat leaf POD activity along with the increase of salt concentration and stress time present the changing trend of lowering after increasing first and reaches the maximum when dealing with 1 d but with no significant difference between varieties; this may be at the beginning of the adversity with POD and varieties of instantaneous reaction related to stress after 4 d significant difference between varieties. This reflects the difference of salt tolerance and self-regulation ability among varieties.

MDA is an important product of membrane lipid peroxidation decomposition, and its content can reflect the degree of membrane peroxidation damage and crop resistance to stress conditions. The process of membrane lipid peroxidation can be enhanced in plants under adverse conditions such as low temperature, drought, and high salinity. It was found in this study that under salt stress, MDA content in wheat leaves of various varieties increased with the increase of salt concentration and stress time to different degrees. QM 6 and DK 961 varieties had a small increase and a mild degree of membrane damage, while JM 22 and QF 1 varieties had a rapid increase in MDA content and a serious degree of membrane damage.

Soluble sugars and soluble proteins can maintain enzymatic activity in the salt solution. When wheat is under stress during growth, the content of soluble sugar in the body will accumulate a lot. Soluble sugar ginseng plays a key role in cell osmoregulation. The increase in soluble sugar can maintain cell turgor pressure, reduce the osmotic potential of the plant body to maintain the plant's required moisture in adversity, and improve the plant's adaptability; this study found that under salt stress, the varieties of wheat leaf soluble sugar content with the increase of salt concentration and stress time showed varying degrees of increase. Compared with JM 22 and QF 1, QM 6 and DK 961 had stronger salt tolerance, and their soluble sugar content increased and accumulated more. The results showed that under salt stress, the content of soluble protein in leaves of all varieties decreased with the increase of salt concentration and stress time to different degrees. JM 22 and QF 1 showed a greater decrease in soluble protein, while the content of soluble protein in the other two varieties was relatively higher. The role of proline is to balance the high concentration of salts in the vacuole and prevent cytoplasmic dehydration. Although the accumulation of proline in plant cells under salt stress is universal, there are still diametrically opposite conclusions about its physiological significance. Some studies suggest that the accumulation of proline under salt stress can be used as an indicator of stress damage. This may be related to the experimental environment and experimental treatment conditions. The results showed that the varieties of wheat leaf proline content under salt stress along with the increase of salt concentration and stress time in different ratios increased, but compared with other indexes' determination results, 4 d after stress, there was significant difference between varieties, salt-tolerant varieties of green wheat, DE 6, 961 growth ratio is larger, and the accumulation of proline content is more. These results indicated that the accumulation of free proline content was an effective measure to improve salt tolerance of wheat.

Root growth and vigor directly affect shoot growth and yield. Root vigor is one of the main indexes to measure root function. Wheat roots can resist salt stress only when they have strong vitality. Root activity reflects the growth capacity and activity level of plant roots. Under adverse conditions, it will lead to the decline of plant root vigor. The root activity reached the maximum value one day after stress and then decreased rapidly. This may be because wheat roots are very sensitive to salt stress, initially increased by self-regulation at the initial stage of stress, but could not be maintained for a long time. With the extension of stress time, the root activity began to decline. However, there were significant differences among varieties, which were most significant at 240 mmol/L salt concentration and stress for 7 days. The root activity of salt-tolerant varieties QM 6 and DK 961 was significantly higher than that of JM 22 and QF 1 by about 3-4 times. Increased root activity was the key factor for QM 6 and DK 961 varieties to resist salt stress.

This study showed that all the abovementioned seven traits could be used as research indexes for the wheat seedling stage, especially the root vigor index, which had a strong screening value for salt tolerance of wheat varieties. The salinity tolerance of QM 6 and DK 961 at the seedling stage was significantly higher than that of JM 22 and QF 1. However, the action mechanism of the abovementioned 7 specific physiological and biochemical indicators still needs to be further studied using molecular technology (as demonstrated in Figure 4).

### 5.3. Effects of Salt Stress on Absorption Ion Partitioning in Wheat at the Seedling Stage

Under salt stress, the concentration of salt ions is too large, and a large amount of Na^+^ and Cl^−^ are accumulated, which can easily cause ion toxicity. If the concentration of salt in plants exceeds or greatly exceeds the range that plants can bear, it will result in plant salt damage. Therefore, the direct consequence of excessive salt accumulation is ion toxicity. On the premise of satisfying cell osmoregulation and ion requirement, the salt concentration of the aboveground part is kept relatively low. This study found that under salt stress, the Na^+^ content in the shoot and root of wheat under all treatments showed a sharply increasing trend, and the amplitude increased with the increase of salt concentration and stress time. Without salt stress, there was no significant difference in Na^+^ content among different treatments. The increase of Na^+^ content in the shoot of salt-tolerant varieties QM 6 and DK 961 was smaller than that of JM 22 and QF 1. However, the variation of Na^+^ content in root cultivars was significantly different from that in the shoot, with the most significant increase in QM 6 and DK 961. From the perspective of sodium limiting ability, the Na^+^ limiting ability of wheat treated with 80 mmol/L salt stress was slightly decreased, except for JM 22 and QF 1 at 7 days of salt stress; the other varieties showed an evident upward trend at this concentration, which may be due to the increase of Na^+^ limiting the ability of wheat under low salt concentration. However, with the salt concentration of 160 mmol/L, only QM 6 and DK 961 showed higher Na^+^ limiting ability than the control, indicating that they still maintained high salt tolerance at this concentration. Under 240 mmol/L NaCl stress, the Na^+^ limiting ability of all cultivars was lower than that of the control treatment, but JM 22 and QF 1 had a significant decrease compared with QM 6 and DK 961. Under salt stress, there were significant differences among the treatments, and QM 6 and DK 961 showed strong Na^+^ limiting ability, which induced high salt tolerance.

To a certain extent, Ca^2+^ can eliminate or alleviate the inhibition of salt on plant growth and enhance plant salt tolerance. It was found that under salt stress, salt ions inhibited the absorption of Ca^2+^ in plants, resulting in the reduction of Ca^2+^ content, the destruction of the balance of Na^+^/Ca^2+^ ratio, the destruction of plasma membrane permeability, and the increase of plasma membrane permeability. In this study, the aboveground and root Ca^2+^ contents of wheat decreased under salt stress in all treatments, and the decrease increased with increasing salt concentration and stress time and the decrease in roots was slightly greater than the decrease in aboveground compared with JM (jimai) 22 and QM (qingmai) 1. The aboveground and root Ca^2+^ contents of QM (qingmai) 6 and DK (dekang) 961 decreased less with increasing salt concentration and stress time and maintained relatively high Ca^2+^ contents. As the content of Ca^2+^ decreased and the content of Na^+^ increased significantly after salt stress, the Ca^2+^/Na^+^ ratio in the shoot and root of wheat in all treatments showed a sharp decreasing trend, and the decreased amplitude increased with the increase of salt concentration and stress time. Under salt stress, the reduction of Ca^2+^/Na^+^ in the shoot of QM 6 and DK 961 was smaller than that of JM 22 and QF 1, while the change of Ca^2+^/Na^+^ among root cultivars was consistent with that of the shoot under salt stress (Figure 5).

Previous studies have found that in a high Na^+^ plant environment, K^+^ is often critically absent, which is caused by the competition between K^+^ and Na^+^ [22]. There are two main ways to maintain high K^+^ in wheat: increasing the absorption of K^+^ and decreasing the affluence of K^+^ because K^+^ plays a crucial role in the physiological activity of wheat salt tolerance, and its content is an important index to measure wheat salt tolerance. Therefore, by reducing the uptake of Na^+^ or inhibiting the upward transport of Na^+^, the normal physiological function of shoot mesophyll cells can be maintained, and the photosynthetic and other physiological and biochemical abilities can be maintained, to improve the salt tolerance of wheat. The results of this study were consistent with the study of Liran Shi. K^+^ content in the shoot and root of wheat was decreased in all treatments, but the K^+^ content in the shoot decreased less than that in the root. Compared with QM 6 and DK 961, the K^+^ content in the shoot and root of JM 22 and QF 1 decreased slightly with the increase in salt concentration and stress time. Because the content of K^+^ decreased and the content of Na^+^ increased significantly after salt stress, the K^+^/Na^+^ ratio in the shoot and root of wheat in all treatments showed a sharp declining trend, and the decreased amplitude increased with the increase of salt concentration and stress time. Under salt stress, the reduction of K^+^/Na^+^ in the shoot of QM 6 and DK 961 was smaller than that of JM 22 and QF 1, which was necessary to control the excessive imbalance of ion ratio and maintain high salt tolerance. There were significant differences among cultivars. Under salt stress, the changes of K^+^/Na^+^ in root cultivars were the same as those in the shoot, but the difference was small. There was no significant difference among varieties (demonstrated in Figure 6).

With the increase in NaCl concentration and stress time, K^+^ and Ca^2+^ in the shoot and root decreased, Na^+^ increased to varying degrees, and K^+^/Na^+^ showed a sharp downward trend. The decrease of Ca^2+^ and K^+^ content in the root of wheat was slightly larger than that in the shoot, but the increase of Na^+^ content in the shoot was smaller than that in the root. In the salt-tolerant varieties QM 6 and DK 961, K^+,^ and Ca^2+^ decreased less than that of JM 22 and QF 1, and the Na^+^ accumulation was lower in shoot than that of JM 22 and QF 1; but the case was the opposite in root, and QM 6 and DK 961 had higher sodium limiting ability. This indicates that limiting Na^+^ transport to shoot for accumulating and maintaining high K^+^/Na^+^ is one of the strategies for wheat salt tolerance (demonstrated in Figure 7).

### 5.4. Effects of Salt Stress on Photosynthetic Characteristics of Wheat after Anthesis

Photosynthesis is the key factor for plants to accumulate nutrients to complete the whole growth and development. The damage to photosynthesis will directly affect another physiological metabolism of plants. The results showed that the chlorophyll content, leaf area index, net photosynthetic rate, stomatal conductance, and transpiration rate of wheat under salt stress decreased compared with the control treatment, and gradually decreased with the increase of salt concentration, and there were significant differences among varieties and different salt concentration treatments. Under salt stress, the intercellular carbon dioxide concentration in flag leaves of wheat increased compared with that of the control and gradually increased with the increase of salt concentration. There were significant differences among varieties and different salt concentration treatments. The chlorophyll content and leaf area index (LAI) were the basic conditions to ensure the smooth progress of photosynthesis. In the control treatment, the chlorophyll content and LAI of JM 22 were higher than those of QM 6, and there was a significant difference between the two varieties in the salt concentration above 3‰, and the content reduction of QM 6 was significantly lower than that of JM 22. Stomatal conductance is an important index reflecting the gas exchange capacity of leaves, which directly affects net photosynthesis. The higher stomatal conductance and transpiration rate of JM 22 under the control treatment may be some of the factors contributing to its higher transpiration rate. Under salt stress, the stomatal conductance and transpiration rate of JM 22 were significantly decreased, and the intercellular carbon dioxide concentration was significantly increased, which may be an important reason for its weak salt tolerance. Under salt stress, QM 6 had a small decrease in stomatal conductance and a small increase in intercellular carbon dioxide concentration. Maintaining a relatively high transpiration rate could effectively use soil water, so the decrease in net photosynthetic rate was low and the net photosynthetic rate was high. The results provided a guarantee for maintaining high photosynthesis under salt stress conditions and laid a foundation for QM 6 to obtain stable and high yield under saline-alkali soil conditions.

As can be seen from Figure 8, according to the experiment, the chlorophyll content, leaf area index, stomatal conductance, and transpiration rate of wheat all decreased, and the intercellular carbon dioxide concentration increased, which inhibited the photosynthesis of wheat and reduced the net photosynthesis of wheat. Compared with JM 22, the salt stress had relatively little effect on the photosynthetic characteristics of QM 6, but the salt resistance ability was stronger, especially in QM 6, which could maintain high photosynthetic characteristics under salt stress, which was the key factor for its high and stable yield on saline-alkali soil. The effects of salt stress on photosystem reaction, photosynthetic energy, and electron transport and conversion need to be further studied.

### 5.5. Effect of Salt Stress Treatment on Wheat Yield

Crop yield and its constituent factors under stress are important manifestations of cultivar stress resistance. Salt stress not only affects seed germination, seedling emergence, and photosynthetic capacity of wheat but also causes the decline of dry matter production and accumulation capacity of wheat, resulting in reduced yield. In this study, it was found that under salt stress, both varieties had different degrees of yield reduction compared with the control. Compared with the varieties, although JM (jimai) 22 maintained a higher thousand grain weight, its spike number and spike number per hectare decreased more than that of QM (qingmai) 6, especially the spike number per hectare decreased the most, and salt stress had a greater effect on intervarietal tillering spike rate, which in turn affected wheat yield and led to yield reduction. QM 6, under salt stress, can still maintain a high population number and panicle number per mu, which is the key factor for its high and stable yield on saline-alkali soil (demonstrated Figure 9).

Salt stress affected wheat dry matter formation and accumulation, affected grain number per ear and 1000-grain weight, and seriously affected wheat tiller and panicle number, resulting in wheat yield reduction. Compared with JM 22, the salt stress had less effect on the yield of QM 6, but the salt resistance ability was stronger, especially in QM 6, which could maintain a higher number of panicles per mu under salt stress, which was another key factor for its high and stable yield on saline-alkali soil.

## 6. Conclusion

The physiological and biochemical indexes of different salt-tolerant wheat varieties under salt stress were affected to different degrees. The changes in physiological and biochemical indexes in salt-tolerant wheat varieties were moderate, while salt-sensitive wheat varieties had bigger changes. In this article, through comprehensive utilization of germination and seedling indoor test morphological indexes, physiological and biochemical index, and output index combined with the appraisal evaluation specification of wheat salt resistance, different types of salt tolerance in wheat in the middle and lower reaches of the Yangtze River in Shandong province; a collection of 100 wheat varieties and 11 salt-resistant wheat varieties planted over a large area is divided into three levels:e strong, medium salt resistance, and weak salt resistance.

The results showed that there were significant differences in salt tolerance among the 100 wheat varieties at the germination stage. Among them, three varieties, YM (Yangmai) 25, YM (Yangmai) 24, and EM (Emai) 25, had the strongest salt tolerance at the germination stage, reaching the level of the salt tolerance variety DK 961, and the salt tolerance was in the first level, while NM 17, NM 23, and other 21 varieties reached the level of the salt tolerance. These 24 varieties with strong salt tolerance at the germination stage can be used to screen the salt tolerance of wheat planted in saline soil of Jiangsu coastal beach. DK 961 and QM 6 showed high salt tolerance. YN 24, LX 99, QF 1, TN 18, and SN 21 showed moderate salt tolerance to salt stress. YN 21, LM21, YN 836, and JM 22 were salt-sensitive types. Further study found that wheat 22 was suitable for low salinity, and water is sufficient for a dramatic increase in production conditions, suitable under the condition of low salt and high fertilizer; green wheat 6 maintains a relatively optimal physiological state under salt stress conditions, and its metabolism, photosynthetic capacity, and salt tolerance ability is strong; its tolerance in the high middle and low salt stress conditions is more outstanding. It is an excellent cultivar adapted to salinized areas, so QM 6 should be planted mainly in salinized areas in Shandong province and its surrounding areas. The chlorophyll content, leaf area index, stomatal conductance, and transpiration rate of wheat were decreased, and the intercellular carbon dioxide concentration was increased, which inhibited the photosynthesis of wheat and reduced the net photosynthesis of wheat. Compared with JM 22, the salt stress had relatively little effect on the photosynthetic characteristics of QM 6, but the salt resistance ability was stronger, especially QM 6, which could maintain high photosynthetic characteristics under salt stress, which was the key factor for its high and stable yield on saline-alkali soil.

## Figures and Tables

**Figure 1:** Salt stress test chart of wheat.

**Figure 2:** Salt tolerance grading diagram.

**Figure 3:** Local data map of germination rate, coleoptile length, root length, and root number.

**Figure 4:** Map of osmotic regulatory substances and root activity index of wheat seedlings (stress day 7).

**Figure 5:** Effects of different salt stress treatments on the dynamic changes of Ca^2+^/Na^+^ in winter wheat (7 d).

**Figure 6:** Effects of different salt stress treatments on the dynamic changes of K^+^/Na^+^ in winter wheat (7 d).

**Figure 7:** Effects of different salt stress treatments on the dynamic changes of the ability to limit Na^+^ content in winter wheat (7 d).

**Figure 8:** Effects of salt stress on photosynthetic characteristics of flag leaves after anthesis of wheat.

**Figure 9:** Effects of different salt stress treatments on grain yield and yield components.

**Table 1:** 100 copies of the middle and lower reaches of the Yangtze River's wheat varieties.

No	Var.	From
1	NM3	1
2	NM 6	1
3	NM 7	1
4	NM 8	1
5	NM 9	1
6	NM 10	1
7	NM 11	1
8	NM 12	1
9	NM 13	1
10	NM 14	1
11	NM 15	1
12	NM 16	1
13	NM 17	1
14	NM 18	1
15	NM 19	1
16	NM 20	1
17	NM 21	1
18	NM 22	1
19	NM 23	1
20	NM 24	1
21	SK1	1
22	SK2	1
23	SX3	1
24	SX4	1
25	SX5	1
26	SX6	1
27	YM5	1
28	YM6	1
29	YM158	1
30	YM9	1
31	YM10	1
32	YM11	1
33	YM12	1
34	YM13	1
35	YM14	1
36	YM15	1
37	YM16	1
38	YM17	1
39	YM18	1
40	YM19	1
41	YM20	1
42	YM21	1
43	YM22	1
44	YM23	1
45	YM24	1
46	YM25	1
47	YGB1	1
48	YRM2	1
49	YRM3	1
50	YRM4	1
51	YRM5	1
52	ZM5	1
53	ZM6	1
54	ZM8	1
55	ZM168	1
56	ZM9	1
57	ZM10	1
58	ZM11	1
59	NN06Y86	1
60	SM3	1
61	SM5	1
62	SM188	1
63	SKM1	1
64	HM5	1
65	HM6	1
66	NGB1	1
67	NY1	1
68	EM11	2
69	EM12	2
70	EM14	2
71	EM15	2
72	EM16	2
73	EM17	2
74	EM18	2
75	EM19	2
76	EM21	2
77	EM22	2
78	EM23	2
79	EM24	2
80	EM25	2
81	EM26	2
82	EM27	2
83	EM251	2
84	EM352	2
85	EM580	2
86	EM596	2
87	HM8	2
88	HM12	2
89	XM25	2
90	XM55	2
91	WM23	3
92	WM26	3
93	WM27	3
94	WM32	3
95	WM35	3
96	WM42	3
97	WM43	3
98	WM54	3
99	LX22	3
100	AN92484	3

Note. 1 representative from Jiangsu Province; 2 representatives from Hubei Province; 3 representatives from Anhui Province.

## Data Availability

The experimental data used to support the findings of this study are available from the corresponding author upon request.
